# Anti-inflammatory Mechanism of Action of Benzoylmesaconine in Lipopolysaccharide-Stimulated RAW264.7 Cells

**DOI:** 10.1155/2022/7008907

**Published:** 2022-07-13

**Authors:** Changkai Zhou, Jing Gao, Haijun Qu, Long Xu, Bin Zhang, Qie Guo, Fanbo Jing

**Affiliations:** ^1^Department of Pharmacy, The Affiliated Hospital of Qingdao University, Qingdao, Shandong, China; ^2^Department of Pharmacy, The Third People's Hospital of Qingdao, Qingdao, Shandong, China

## Abstract

**Background:**

Benzoylmesaconine (BMA), the most abundant monoester alkaloid in *Aconitum* plants, has some biological activities and is a potential therapeutic agent for inflammation-related diseases. However, the potential anti-inflammatory mechanisms of BMA have not been clarified.

**Purpose:**

This study aimed to investigate the underlying molecular mechanisms of the anti-inflammatory action of this compound using lipopolysaccharide (LPS)-activated RAW264.7 macrophages.

**Methods:**

The release of pro-inflammatory cytokines and mediators were detected by nitric oxide (NO) assays, reactive oxygen species (ROS) assays, and enzyme-linked immunosorbent assays (ELISA) in LPS-activated RAW264.7 macrophage cells. Quantitative real-time PCR was used to measure the gene expression of interleukin (IL)-1*β*, tumor necrosis factor (TNF)-*α*, IL-6, inducible nitric oxide synthase (iNOS), and cyclooxygenase-2 (COX-2). Cell viability was determined using a cell counting kit-8 (CCK-8) assay. The expression of iNOS, COX-2, mitogen-activated protein kinase (MAPK), and nuclear factor-*κ*B (NF-*κ*B)-related proteins were detected by western blot, and nuclear translocation of p65 was observed by immunofluorescence.

**Results:**

BMA significantly decreased the production of IL-1*β*, IL-6, TNF-*α*, PGE_2_, NO, and ROS and inhibited the protein and mRNA levels of COX-2 and iNOS in LPS-activated RAW264.7 macrophages. Moreover, LPS-induced phosphorylation of I*κ*B*α*, JNK, p38, and ERK; degradation of I*κ*B*α*; and nuclear translocation of p65 were significantly suppressed by BMA treatment.

**Conclusion:**

These findings demonstrate that the anti-inflammatory effect of BMA was through the suppression of the NF-*κ*B and MAPK signaling pathways and that it may be a therapeutic agent targeting specific signal transduction events required for inflammation-related diseases.

## 1. Introduction

Inflammation is a defense response of the body initiated by tissue injury or pathogen invasion [1, 2]. However, the abnormal or uncontrolled inflammatory response has harmful effects on the host and can cause numerous diseases, including arthritis, cancer, atherosclerosis, and obesity [3]. Macrophages are important immune cells whose activation is commonly accompanied by inflammation and are involved in various disease processes to regulate immune response [1]. During inflammatory response processes, macrophage activation triggered by LPS simulation leads to the activation of specific signaling cascades and the release of pro-inflammatory cytokines and mediators, including IL-1*β*, TNF-*α*, PGE_2_, and NO [4, 5].

Transmembrane proteins expressed on some immune cells, like Toll-like receptors (TLRs), affect the activation of innate immune cells [6]. LPS is an important structural component of the outer membrane of Gram-negative bacteria, which can be specifically sensed by TLR4, a member of the TLR family expressed by innate immune cells, like macrophages. Upon LPS recognition, TLR4 undergoes oligomerization and recruits its downstream adaptors through interactions with TIR (Toll-interleukin-1 receptor) domains, which mediate protein-protein interactions between TLRs and signal transduction adaptor proteins, such as MyD88. LPS-induced TLR4 activation can trigger downstream signaling pathways involving both NF-*κ*B and MAPK [7, 8]. The NF-*κ*B pathway plays a key role during the inflammatory response by regulating the transcription of certain genes for growth factors, COX-2, iNOS, and pro-inflammatory cytokines [1, 9, 10]. NF-*κ*B exists in an inactive form, which is a heterotrimer composed of I*κ*B proteins, p65, and p50 in the cytosol in its unstimulated state. LPS-induced inflammatory responses can activate I*κ*B kinase (IKK), leading to I*κ*B phosphorylation and degradation in the ubiquitination pathway, and then NF-*κ*B dissociates from I*κ*B/NF-*κ*B and translocates into the nucleus where NF-*κ*B binds to DNA and subsequently initiates further inflammatory responses and pro-inflammatory gene expression [9, 11, 12].

In addition, the activation of the MAPK family consisting of p38, JNK, and ERK promotes the expression of activator protein-1 (AP-1), a transcription factor closely associated with diverse cellular processes, such as pro-inflammatory cytokine production, cell differentiation, survival, and apoptosis [13]. In activated macrophages, MAPK pathway activation gives rise to the release of various pro-inflammatory mediators during an inflammatory response [14]. Thus, regulation of the MAPK and NF-*κ*B pathways is an effective therapeutic strategy for anti-inflammatory drugs that treat inflammation.

Traditional Chinese medicine, like *Aconitum* plants whose effective components are *Aconitum* alkaloids, have been widely used in orthopedic diseases, such as rheumatoid arthritis (RA), for over two thousand years. Mesaconitine, hypaconitine, and aconitine, belonging to the diester-diterpenoid alkaloid group, possess high levels of human toxicity. BMA (Figure 1), which can be produced by hydrolysis of hypaconitine, possesses some biological activities, including antifungal, antiviral, anti-inflammatory, and analgesic activities [15–17], and its content is higher than the other two monoester-diterpenoid alkaloids, benzoylaconine (BAC) and benzoylhypaconine (BHA), in *Aconitum* plants [18]. Due to its low toxicity, considerable pharmacology, and abundance, the current study selected BMA as an anti-inflammatory drug to investigate its underlying molecular mechanisms.

Although previous studies have indicated that BMA exhibits anti-inflammatory activity, little is known about its underlying molecular mechanisms of regulating inflammatory response, which limits the application of BMA as a therapeutic tool for the treatment of inflammatory diseases. In this study, we assessed the effects of BMA on inflammatory response attenuation via the inhibition of the activation of the MAPK and NF-*κ*B signaling pathways using LPS-activated RAW264.7 macrophages, thus providing new scientific evidence for BMA's efficacy for the treatment of clinical inflammatory disorders.

## 2. Materials and Methods

### 2.1. Materials

RAW264.7 cells and BMA (purity ≥98%) were provided by the Chinese Academy of Sciences (Shanghai, China) and Yousi Scientific Co., Ltd. The NO Assay Kit was acquired from Jiancheng Bioengineering Institute (Nanjing, China). ELISA kits were obtained from Elabscience (Wuhan, China). Anti-p-NF-*κ*B, anti-p-JNK, anti-p-p38, anti-p-ERK1/2, anti-NF-*κ*B, anti-JNK, anti-p38, and anti-ERK1/2 antibodies were purchased from Abcam (Cambridge, UK). Anti-p-I*κ*B*α* and anti-I*κ*B*α* antibodies were obtained from Affinity Bio Reagents (Golden, CO, USA). LPS from *Escherichia coli* and TPCK (NF-*κ*B inhibitor) were obtained from Sigma (St. Louis, MO, USA). CCK-8, SP600125 (JNK inhibitor), SB202190 (p38 MAPK inhibitor), and U0126 (ERK inhibitor) were obtained from Medchem Express (St. Louis, MO, USA). Trizol and phenylmethanesulfonyl fluoride (PMSF) were acquired from Ambion (CA, USA) and Aladdin (Shanghai, China). An RNA extraction kit, HiScript II *Q* Select RT SuperMix, and SYBR Green Master Mix were provided by VAZYME (Nanjing, China). ROS Assay Kits, BCA Protein Assay Kits, radioimmunoprecipitation assay (RIPA), phosphatase inhibitor cocktail, and enhanced chemiluminescence (ECL) substrate were acquired from Beyotime (Shanghai, China). PVDF membranes were obtained from Millipore (Billerica, MA, USA). Fetal bovine serum (FBS) and Dulbecco's modified Eagle's medium (DMEM) were obtained from Gibco (Grand Island, NY).

### 2.2. Cell Culture

Cells were cultured in DMEM containing 10% FBS at 37°C in a 5% CO_2_ moist atmosphere. After pretreatment with the indicated concentrations of BMA for 1 h, cells were stimulated with LPS that had been diluted to 1 *μ*g/mL with a culture medium at different time points.

### 2.3. CCK-8 Assays

Cells were incubated at 1.5 × 10^4^ cells/well in 96-well plates for 24 h and then treated with serial concentrations of BMA (40, 80, or 160 *μ*M) for 1 h with or without 1 *μ*g/mL LPS for 24 h in triplicate. Finally, 10 *μ*L of CCK-8 was added to each well. After incubation for another 24 h at 37°C, the absorbance was detected at the wavelength of 450 nm using a FlexStation 3 microplate reader (Molecular Devices, CA, USA).

### 2.4. ROS Assays

To detect ROS levels, cells were treated with BMA (40, 80, or 160 *μ*M) for 1 h before being stimulated with LPS (1 *μ*g/mL) for 24 h. Then cells were incubated with DCFH-DA (10 *μ*M) for 20 min after the medium was removed. After sufficient washing, the ROS levels were measured using an Olympus BX53 fluorescence microscope (Olympus, Japan) with excitation and emission wavelengths of 488 nm and 525 nm, respectively.

### 2.5. ELISA Assays

After pretreatment with BMA (40, 80, or 160 *μ*M) for 1 h, cells were stimulated by LPS (1 *μ*g/mL) for another 24 h in DMEM to measure IL-1*β*, TNF-*α*, IL-6, and PGE_2_ levels. ELISA kits (Elabscience, Wuhan, China) were used to determine the production of pro-inflammatory cytokines according to the manufacturer's instructions.

### 2.6. qRT-PCR

Macrophages were incubated in 96-well plates at 1.5 × 10^4^ cells/well for 24 h and then treated with serial concentrations of BMA (40, 80, or 160 *μ*M) for 1 h before LPS (1 *μ*g/mL) stimulation for 24 h. Total RNA was extracted with an RNA extraction kit and transformed to cDNA using HiScript II *Q* Select RT SuperMix according to the manufacturer's protocol. Specific primer sequences used for PCR were as follows: TNF-*α* (sense: GCCTATGTCTCAGCCTCTTCT, antisense: TTGTGAGTGTGAGGGTCTGG); IL-1*β* (sense: TCAGGCAGGCAGTATCACTC, antisense: AGCTCATATGGGTCCGACAG); IL-6 (sense: CACAGAGGATACCACTCCCAACAGA, antisense: ACAATCAGAATTGCCATTGCACAAC); iNOS (sense: CACCTTGGAGTTCACCCAGT, antisense: ACCACTCGTACTTGGGATGC); COX-2 (sense: AGGTCATTGGTGGAGAGGTG, antisense: CCTGCTTGAGTATGTCGCAC); and *β*-actin (sense: CACGATGGAGGGGCCGGACTCATC, antisense: TAAAGACCTCTATGCCAACACAGT). Relative mRNA concentrations were quantitated using SYBR Green Master Mix on an ABI QuantStudio 6 Real-Time PCR System. The 2^−ΔΔCt^ method was used to analyze data for relative gene expression.

### 2.7. Western Blot Analysis

Macrophages were incubated with or without LPS (1 *μ*g/mL) in the presence of serial concentrations of BMA (40, 80, or 160 *μ*M). Then, ice-cold phosphate-buffered saline (PBS) was used to wash these macrophages three times, and phosphatase inhibitor cocktail and RIPA buffer supplemented with PMSF were used to extract whole-cell proteins. Subsequently, a BCA protein assay was used to measure the total protein concentration of each lysate. 40 *μ*g of protein was transferred onto PVDF membranes, and each immunoblot was then blocked for 2 h with 10% nonfat milk in Tris-buffered saline Tween 20 (TBST). Subsequently, membranes were incubated with primary rabbit antibodies at 4°C and washed with TBST five times, followed by incubation for 2 h with goat anti-rabbit IgG HRP at room temperature. Finally, membranes were analyzed using an ECL substrate.

### 2.8. Immunofluorescence Assays

Cells were treated with BMA (160 *μ*M) for 1 h before stimulation by LPS (1 *μ*g/mL) for 0.5 h and then washed twice with PBS. 4% paraformaldehyde and 0.5% Triton *X*-100 were used to fix and permeabilize cells for 0.5 h, respectively. After blocking with normal goat serum, cells were incubated overnight at 4°C with primary antibodies against NF-*κ*B p65. After washing with PBS, Cy3-labeled goat anti-rabbit IgG was used as a secondary antibody for 0.5 h. A BX53 fluorescence microscope (Olympus, Japan) was used to visualize cells stained with 4′,6-diamidino-2-phenylindole (DAPI) after the removal of the secondary antibody and sufficient washing.

### 2.9. NO Assay

Griess reagent was used to determine the NO levels in activated macrophages. SP600125, TPCK, SB202190, or U0126 was administered to macrophages separately with or without BMA (160 *μ*M) for 1 h, and then cells were stimulated by LPS (1 *μ*g/mL) for 24 h. Subsequently, 50 *μ*L of medium from each was mixed with an equal volume of 50 *μ*L Griess reagent in 96-well plates and the reaction was incubated for 5 min. After the supernatant was collected, the NO levels in activated RAW264.7 cells were determined using an NO Assay Kit, and the absorbance at 540 nm was measured using a microplate reader.

### 2.10. Statistical Analysis

Data were analyzed using SPSS v22 software (IBM, Armonk, NY, USA) and are presented as mean ± SD from at least triplicate experiments. One-way ANOVA was used to assess the statistical differences between groups. A *P* < 0.05 was considered to be statistically significant.

## 3. Results

### 3.1. Effect of BMA on Cell Viability

A CCK-8 assay was used to examine the potential cytotoxicity of BMA in RAW264.7 cells before investigating the molecular mechanisms of its anti-inflammatory action. The percentages of cell viability were from 96.30% to 103.07%, indicating that BMA was nontoxic to macrophages below 160 *μ*M after a 24-h treatment (Figure 2). Therefore, BMA was used at concentrations of 40, 80, and 160 *μ*M for subsequent experiments.

### 3.2. BMA Inhibited the Production of TNF-*α*, IL-1*β*, and IL-6 in LPS-Activated RAW264.7 Macrophages

The excessive activation of macrophages by LPS stimulation leads to a significant release of pro-inflammatory cytokines. The production of TNF-*α*, IL-1*β*, and IL-6 were significantly upregulated with LPS treatment compared to control cells. 160-*μ*M BMA exerted an inhibitory effect on the production of pro-inflammatory cytokines and decreased their levels to 89.42, 56.56, and 55.15 pg/mL, respectively (Figures 3(a)–3(c)). To find out whether BMA could regulate the transcriptional levels of pro-inflammatory cytokines, the mRNA expression of TNF-*α*, IL-1*β*, and IL-6 was measured. Compared with the LPS-treated group, the mRNA levels of TNF-*α*, IL-1*β*, and IL-6 were significantly reduced by BMA treatment in LPS-activated RAW264.7 macrophages (Figures 3(d)–3(f)). Taken together, these results indicated that the anti-inflammatory activity of BMA function through suppressing pro-inflammatory cytokine expression.

### 3.3. BMA Inhibited the Production of ROS, PGE_2_, and NO in LPS-Activated RAW264.7 Macrophages

As shown in Figure 4(a), we observed that BMA markedly inhibited the LPS-induced production of ROS in a dose-dependent manner. Meanwhile, we used ELISA to examine the effects of BMA on the production of PGE_2_. LPS stimulation remarkably elevated PGE_2_ levels as compared with nontreated cells, whereas treatment with BMA effectively suppressed this elevation in a dose-dependent manner (Figure 4(b)). As shown in Figure 4(c), the NO production was markedly upregulated in LPS-stimulated RAW264.7 cells compared with control cells, whereas 160-*μ*M BMA treatment significantly decreased the NO level by 58.92%. To further investigate the association between the MAPK and NF-*κ*B pathways and the anti-inflammatory effect of BMA, we combined inhibitors, including TPCK, U0126, SP600125, and SB202190, with BMA in subsequent experiments. There was no significant difference in LPS-induced NO production between combined treatment groups and the BMA treatment group, indicating that the inhibitory effect of BMA on inflammatory response might be related to the suppression of the NF-*κ*B and MAPK pathways.

### 3.4. BMA Inhibited LPS-Induced COX-2 and iNOS Protein and mRNA Expression in RAW264.7 Macrophages

COX-2 and iNOS have been demonstrated to be the corresponding synthases of PGE_2_ and NO, respectively [3, 19]. We measured the protein and mRNA expression of COX-2 and iNOS to investigate whether BMA inhibited the production of PGE_2_ and NO through suppression of their synthases. Our results showed that the protein and mRNA expression levels of COX-2 and iNOS were upregulated in LPS-activated RAW264.7 macrophages. However, compared with the LPS-stimulated group, treatment with BMA significantly decreased COX-2 and iNOS levels in a dose-dependent manner (Figure 5), suggesting that the decreased production of PGE_2_ and NO were associated with the inhibition of COX-2 and iNOS expression, respectively.

### 3.5. BMA Inhibited the Activation of the NF-*κ*B Pathway in LPS-Activated RAW264.7 Macrophages

NF-*κ*B, as a key transcription factor that regulates the gene expression of pro-inflammatory cytokines and mediators, is activated by inflammatory agents such as LPS [20]. To investigate this potential mechanism of attenuation of inflammatory responses, we assessed the effect of BMA on LPS-induced activation of the NF-*κ*B pathway in RAW264.7 macrophages. Phosphorylation and nuclear translocation of NF-*κ*B p65 were triggered by LPS stimulation, while protein levels of p65 in the nucleus and its phosphorylation were significantly inhibited by BMA treatment in a dose-dependent manner (Figures 6(a), 6(b), and 6(e)). Moreover, as shown in Figure 6(f), the results of immunofluorescence assays suggested that BMA strongly suppressed the LPS-induced nuclear translocation of NF-*κ*B p65. Considering that phosphorylation and degradation of I*κ*B*α* is closely related to NF-*κ*B activation, we next investigated whether BMA affected I*κ*B*α* phosphorylation and degradation. Western blot analysis showed that LPS-induced high levels of I*κ*B*α* phosphorylation and degradation were significantly decreased by BMA treatment in a dose-dependent manner (Figures 6(c) and 6(d)). Taken together, the present study indicated that LPS-induced inflammatory responses in activated macrophages could be attenuated by suppressing NF-*κ*B signaling activation.

### 3.6. BMA Inhibited Protein Expression of the MAPK Pathway in LPS-Activated RAW264.7 Macrophages

LPS stimulation also leads to MAPK signaling pathway activation, causing pro-inflammatory cytokine overproduction and excessive inflammatory response in RAW264.7 macrophages [21]. To further study the potential mechanism of attenuating inflammatory responses, we examined whether BMA affected protein expressions of MAPK pathway proteins in LPS-activated RAW264.7 macrophages. As shown in Figure 7, LPS stimulation resulted in high levels of phosphorylated ERK, JNK, and p38 in macrophages, whereas BMA downregulated LPS-induced protein expression of p-ERK, p-JNK, and p-p38 in a dose-dependent manner. The above results implied that the mechanism of attenuating the inflammatory response exerted by BMA might be linked to the regulation of the MAPK signal pathway in LPS-induced RAW264.7 macrophages.

## 4. Discussion

Inflammation, as a protective response, can protect organisms when fungi, viruses, or bacteria invade the body [22]. During the development of inflammation, macrophage activation can release various pro-inflammatory cytokines and mediators, the levels of which are believed to be an indicator of the degree of inflammation. Therefore, anti-inflammatory agents are generally searched through inhibiting the overproduction of cytokines and mediators. Although nonsteroidal anti-inflammatory drugs (NSAIDs) are traditional therapeutic drugs for inflammatory diseases, their long-term use can cause some side effects [23, 24]. Thus, seeking safer and more effective anti-inflammatory agents has great significance for the treatment of clinical inflammatory disorders. Compared with NSAIDs, some alkaloid components in herbal plants exhibit anti-inflammatory activity with less side effects.

*Aconitum* plants are well-known traditional Chinese herbs that contain some active and toxic substances, such as alkaloids. Compared to diester-diterpenoid alkaloids, including hypaconitine, mesaconitine, and aconitine, monoester-diterpenoids have much lower human toxicity. BMA, BAC, and BHA are representative monoester-diterpenoid alkaloids found in *Aconitum* plants, and BMA possesses considerable anti-inflammatory activities and is present at a higher level than the other two monoester-diterpenoid alkaloids—BAC and BHA [25, 26]. However, the potential anti-inflammatory mechanisms of BMA have not been clarified. In our study, we used LPS-stimulated macrophages to study the potential mechanism of the anti-inflammatory activity of BMA and found that it attenuates LPS-induced inflammatory responses via inhibiting the NF-*κ*B and MAPK signaling pathways. These results contribute to providing new support for the use of BMA as a potential anti-inflammatory agent.

Macrophages, as innate immune cells, play a key role in modulating the inflammation processes triggered by LPS simulation during the development of inflammation, leading to the release of pro-inflammatory mediators and cytokines, including PGE_2_, NO, ROS, IL-1*β*, and TNF-*α*, and the activation of specific signaling cascades. The LPS-induced overproduction of cytokines in macrophages has been shown to be involved in the development of inflammation processes. In the present study, we found that BMA attenuated LPS-induced inflammatory responses by suppressing their production in RAW264.7 macrophages. Moreover, we observed a dose-dependent reduction in the iNOS and COX-2 protein expressions, which are key synthases producing NO and PGE_2_, respectively.

During inflammatory response processes, endogenous molecules released by injured tissues and dying cells (DAMPs, damage-associated molecular patterns) and viruses and bacteria (PAMPs, pathogen-associated molecular patterns) can be recognized by innate immune cells, leading to the activation of resident macrophages. TLRs, as pattern recognition receptors, which are abundant in inflammatory tissues of some inflammatory diseases, like RA, can bind to these specific molecules and play a vital role in directing the development of effective immune responses against harmful stimulation [27]. To define the molecular mechanisms by which BMA exerted an inhibitory effect on the production of pro-inflammatory cytokines and mediators, the effects of BMA on LPS-induced activation of the NF-*κ*B and MAPK signaling pathways were further investigated.

TLR4 is considered a vital sensor of LPS simulation and is essential for the activation of downstream NF-*κ*B and MAPK signaling pathways. Activated TLR4 can initiate downstream cell signaling through MyD88-dependent and MyD88-independent (TRIF-dependent) pathways [28], and the TLR4/MyD88/NF-*κ*B pathway has been reported to be one of the most essential signaling pathways in the regulation of inflammation [29]. Moreover, NF-*κ*B plays a vital role in regulating the transcription of numerous pro-inflammatory mediators and cytokines during the inflammatory process [29, 30]. In our study, we found that BMA suppressed the activation of the NF-*κ*B signaling pathway in LPS-activated macrophages. NF-*κ*B exists in an inactive form with I*κ*B, a binding partner and inhibitory protein of NF-*κ*B, in nonactivated macrophages [31, 32]. LPS stimulation significantly influences the inhibitory effect of I*κ*B on NF-*κ*B, and then I*κ*B dissociates from this complex and rapidly degrades in the cytosol. NF-*κ*B translocates to the nucleus and binds to specific DNA sites after it separates from these complexes, which initiates the transcription of pro-inflammatory mediators and cytokines during inflammatory processes [33, 34]. In this study, we found that pretreatment with BMA markedly inhibited the phosphorylation and degradation of I*κ*B*α*. At the same time, immunofluorescence and western blot results showed that LPS-induced p65 nuclear translocation was blocked by BMA, demonstrating that the reduction of pro-inflammatory mediator and cytokine expression might occur via inhibiting the activation of the NF-*κ*B signaling pathway.

JNK, p38, and ERK are three main members of the MAPK family in mammals, which play a critical role in inflammation and participate in the activation of some inflammation-related genes encoding inflammatory cytokines. LPS stimulation leads to the activation of p38, JNK, and ERK through threonine residues and tyrosine phosphorylation. In this study, we investigated whether BMA had an influence on MAPK activation and we found that BMA treatment suppressed LPS-induced phosphorylation of p38, JNK, and ERK in a dose-dependent manner in activated RAW264.7 macrophages, indicating that BMA was also an effective inhibitor of the MAPK signaling pathway. However, in our initial experimental design, we did not add inhibitors of the MAPK or NF-*κ*B signaling pathways to further confirm the effect of BMA on these two pathways in a mechanistic manner. Meanwhile, how BMA regulates upstream adaptor proteins of MAPK and NF-*κ*B in this macrophage model stimulated by LPS, such as the protein TAK1, is not explored. Both of these are crucial topics for further research in the future. Similar to our previous findings [35], results from other current research suggest that monoester-diterpenoid alkaloids in *Aconitum* plants like BMA, BAC, and BHA can attenuate inflammatory responses, probably through the same mechanism.

In conclusion, our results facilitate a better understanding of the molecular mechanism of BMA in LPS-activated RAW264.7 macrophages, and we provide novel evidence that BMA exerts its anti-inflammatory effect through suppressing the activation of the MAPK and NF-*κ*B signaling pathways (Figure 8). Accordingly, our study indicates that BMA may be developed as a new therapeutic candidate to provide protection against inflammatory diseases.

## Figures and Tables

**Figure 1:** Chemical structure of BMA.

**Figure 2:** Effect of BMA on the viability of RAW264.7 cells. Cell viability was assessed after treatment with BMA (40, 80, or 160 *μ*M) for 1 h and stimulated with or without LPS for 24 h. Data are expressed as mean ± SD from three independent experiments. ^#^*P* < 0.05 vs. nontreated group.

**Figure 3:** Effect of BMA on TNF-*α* and IL-1*β* levels in LPS-activated RAW264.7 cells. ((a)–(c)) The levels of TNF-*α*, IL-1*β*, and IL-6 were determined by ELISA after treatment with BMA (40, 80, or 160 *μ*M) for 1 h and stimulation with LPS (1 *μ*g/mL) for another 24 h in LPS-activated RAW264.7 cells. ((d)-(f)) The mRNA levels of TNF-*α*, IL-1*β*, and IL-6 were determined by real-time PCR. Data are expressed as mean ± SD from three independent experiments. ^#^*P* < 0.05 vs. control group, and ^*∗*^*P* < 0.05, ^*∗∗*^*P*  < 0.01 vs. LPS group.

**Figure 4:** Effect of BMA on the production of PGE_2_, NO, and ROS in LPS-activated RAW264.7 cells. (a) Cells were treated with BMA (40, 80, or 160 *μ*M) for 1 h and stimulated with LPS (1 *μ*g/mL) for 24 h The level of ROS was determined using fluorescence microscopy. (b) Cells were treated with BMA (40, 80, or 160 *μ*M) for 1 h and stimulated with LPS (1 *μ*g/mL) for 24 h The level of PGE_2_ production was determined using ELISA. (c) SP600125, TPCK, SB202190, or U0126 was administered to macrophages separately with or without BMA (160 *μ*M) for 1 h, and then cells were stimulated with LPS (1 *μ*g/mL) for 24 h The absorbance at 540 nm was measured using a microplate reader. Data are expressed as mean ± SD from three independent experiments. ^#^*P* < 0.05 vs. control group, and ^*∗*^*P* < 0.05, ^*∗∗*^*P* < 0.01 vs. LPS group.

**Figure 5:** Effect of BMA on the protein expression of COX-2 and iNOS in LPS-activated RAW264.7 cells. ((a)-(c)) Cells were treated with BMA (40, 80, or 160 *μ*M) for 1 h and then stimulated with LPS (1 *μ*g/mL) for 24 h. The level of protein expression was analyzed by western blot, and *β*-actin was used as a loading control. (d) and (e) The mRNA levels of COX-2 and iNOS were determined by real-time PCR. Data are expressed as mean ± SD from three independent experiments. ^#^*P* < 0.05 vs. control group, and ^*∗*^*P* < 0.05, ^*∗∗*^*P* < 0.01 vs. LPS group.

**Figure 6:** Effect of BMA on NF-*κ*B activation in LPS-activated RAW264.7 cells. ((a)-(e)) Cells were treated with BMA (40, 80, or 160 *μ*M) for 1 h and stimulated with LPS (1 *μ*g/mL) for 0.5 h (e) or 24 h (b-d). The protein expression levels were analyzed by western blot. (f) Cells were treated with BMA (160 *μ*M) for 1 h and stimulated with LPS (1 *μ*g/mL) for 0.5 h. A fluorescence microscope was used to obtain images of the nucleus (blue) and NF-*κ*B p65 (red). Data are expressed as mean ± SD from three independent experiments. ^#^*P* < 0.05 vs. control group, and ^*∗*^*P* < 0.05, ^*∗∗*^*P* < 0.01 vs. LPS group.

**Figure 7:** Effect of BMA on MAPK activation in LPS-activated RAW264.7 cells. ((a)-(d)) Cells were treated with BMA (80 or 160 *μ*M) for 1 h and then stimulated by LPS (1 *μ*g/mL) for 24 h. The protein expression levels of ERK, p-ERK, JNK, p-JNK, p38, and p-p38 were analyzed by western blot. Data are expressed as mean ± SD from three independent experiments. ^#^*P* < 0.05 vs. control group, and ^*∗*^*P* < 0.05, ^*∗∗*^*P* < 0.01 vs. LPS group.

**Figure 8:** Schematic representation of the anti-inflammatory mechanisms by BMA in LPS-induced inflammation.

## Data Availability

The data used to support the findings of this study are available from the corresponding author upon request.
